# HMGB3 Targeted by miR-145-5p Impacts Proliferation, Migration, Invasion, and Apoptosis of Breast Cancer Cells

**DOI:** 10.1155/2022/1954099

**Published:** 2022-11-10

**Authors:** Yangying Hu, Deqi Wu, Rong Huang, Zhijie Shi

**Affiliations:** ^1^Department of Thyroid and Breast Diagnosis and Treatment Center, Shulan (Hangzhou) Hospital Affiliated to Zhejiang Shuren University Shulan International Medical College, Hangzhou, Zhejiang 310000, China; ^2^Pathology Department, Shulan (Hangzhou) Hospital Affiliated to Zhejiang Shuren University Shulan International Medical College, Hangzhou, Zhejiang 310000, China

## Abstract

This study focused on the investigation into how HMGB3 works in breast cancer (BC) progression. Firstly, we analyzed the relationship between HMGB3 and BC patients through the TCGA database. We performed qRT-PCR for determining the HMGB3 mRNA level and Western blot for detecting the protein level of HMGB3 in BC cell lines. CCK-8, flow cytometry, transwell, and wound healing assays were utilized to detect the effect of HMGB3 on BC cell phenotypes. Next, the prediction of the binding site shared by miR-145-5p and HMGB3 was performed by the bioinformatics method. The targeting relationship between miR-145-5p and HMGB3 was validated by using dual-luciferase assay. Finally, rescue experiments were employed for assessing the effect of the miR-145-5p/HMGB3 axis on BC cells. HMGB3 was demonstrated to have a high-level expression in BC cell lines and facilitated BC progression. On the contrary, miR-145-5p was shown a low-level expression in BC cell lines, which could target HMGB3. miR-145-5p restrained the proliferation, migration, and invasion of BC cells via inhibiting HMGB3.

## 1. Introduction

As a commonly diagnosed cancer in women, breast cancer (BC) is a big threat to the global women's health [1]. Recently, common clinical therapies of BC include surgery treatment, hormonotherapy, cytotoxic chemotherapy, immunotherapy, and target therapy [2–4]. The patient's survival rate is increased by those therapies, but mortality remains relatively high. The main cause of the death of patients with BC is the metastasis of tumor cells [5]. Hence, continuous exploration into the molecular mechanism of BC progression is indispensable, thus to formulate a more effective treatment.

High mobility group box 3 (HMGB3) is first known as an expressed sequence tag during embryonic development [6, 7]. HMGB3 exerts an indispensable part in DNA recombination, repair, and replication. HMGB3 can modulate gene expression, induce innate immune activity, and regulate the balance between differentiation of hematopoietic stem cells and self-renewal [8, 9]. Besides, HMGB3 is widely involved in regulating pathological states including various cancers, like gastric cancer [10], esophageal cancer [11], and non-small cell lung cancer [12]. Studies demonstrated a high expression level of HMGB3 in BC, and HMGB3 was regarded as a cancer promoter to modulate the development of BC [13, 14]. In BC cells, HMGB3 is upregulated and its silencing impairs cell proliferation *in vitro* and *vivo* [15]. HDAC3 can increase the expression of HMGB3 by downregulating miR-130a-3p and promote the immune escape of BC cells [16]. However, there are scarce studies on the molecular mechanism of HMGB3 involvement in BC and whether HMGB3 exerts a regulatory role in BC progression remains an unanswered question.

MicroRNAs (miRNAs) are pivotal for modulating gene expression. The mechanism of miRNAs is to modulate expression of protein-coding genes by causing mRNA cleavage or translational repression [17]. The role of miRNAs in BC has been investigated [18]. Ashirbekov et al. [19] unveiled the essential part of miR-145-5p in BC which was able to restrain some oncogene expression. miR-145-5p, by targeting SOX2, is able to impede the proliferation of BC cells [20]. But whether there is a connection between the suppressive effect of miR-145-5p and HMGB3 on BC cells has not been revealed.

In this research, the roles of HMGB3 and its upstream regulatory gene miR-145-5p in BC cells were analyzed by bioinformatics analysis and cellular molecular experiments. This study underpins the exploitation of the potential therapeutic targets for BC treatment.

## 2. Materials and Methods

### 2.1. Bioinformatics Analysis

Mature miRNA data (normal: 104, tumor: 1,103) and count data of mRNA (normal: 113, tumor: 1,109) of BC were downloaded from The Cancer Genome Atlas (TCGA) database (https://tcgadata.nci.nih.gov/tcga/tcgaHome2.jsp) (searching keywords were “breast cancer,” “BRCA,” and “Homo sapiens”). After preprocessing them according to PAM50 [21], we obtained Luminal A, Luminal B, Basal, Her2, and nonsubtype samples. Differential expression of HMGB3 in normal breast tissue and BC tissue was determined by *t*-test. Tumor samples were divided on the basis of the median value of HMGB3 expression in all samples or different subtypes of BC, and the “survival” package was used for the conduction of the survival analysis. Afterwards, the Kruskal-Wallis test was employed for analyzing the association between HMGB3 and clinical features and differences of HMGB3 in different BC subtypes.

With “EdgeR” package (∣logFC | >2.0, *P*adj < 0.01), differential analysis was undertaken on miRNAs. To determine the upstream regulator miRNA of HMGB3, starBase (http://starbase.sysu.edu. cn/index.php) and TargetScan (http://www.targetscan.org/vert_72/) databases were applied for prediction. The predicted miRNAs were overlapped with differentially downregulated miRNAs. Pearson correlation analysis was performed on miRNA and HMGB3, and differential expression of miRNA in BC and normal breast tissues was further defined by *t*-test.

### 2.2. Cell Culture and Transfection

The human mammary epithelial cell line MCF-10A (BNCC102049) and BC cell lines MDA-MB-231 (BNCC337894), MDA-MB-468 (BNCC100687), T47D (BNCC339607), and ZR-75-30 (BNCC100125) were all provided by BeNa Culture Collection (China). MCF-10A, MDA-MB-231, T47D, and ZR-75-30 were all treated with 10% FBS-contained (HyClone, USA) DMEM complete medium (Sigma, USA). MDA-MB-468 was maintained in Leibovitz Medium (L15) (Sigma, USA) with 10% FBS. The above cells were placed in a constant temperature incubator at 37°C with 5% CO_2_. miR-mimic, miR-inhibitor, and corresponding negative control (miR-NC) were acquired from GeneChem (China). The following were the sequences: miR-145-5p mimic: 5′-GUCCAGUUUUCCCAGGAAUCCCU-3′, 3′-CAGGUCAAAAGGGUCCUUAGGGA-5′; miR-NC: 5′-UUUGUACUACACAAAAGUACUG-3′, 3′-AAACAUGAUGUGUUUUCAUGAC-5′; miR-inhibitor: 5′-AGGGAUUCCUGGGAAAACUGGAC-3′; inhibitor-NC: 5′-CAGUACUUUUGUGUAGUACAAA-3′; and HMGB3-specific siRNA (si-HMGB3: 5′-GGUCUUCGCCUUGAUUCAUTT-3′, 5′-AUGAUAUAAGGCGAAGACCTT-3′ were procured from GenePharma (China). pcDNA3.1-HMGB3 plasmid that encodes HMGB3 (oe-HMGB3) and empty pcDNA3.1 plasmid (oe-NC) were constructed by GenePharma (China). The 6-well plates were utilized for BC cell (2 × 10^5^ cells/well) seeding. When cells proliferated into 40–50% confluency, the target plasmids (10 *μ*g) or synthesized sequences (50 nM) were transiently transfected for 48 h using Lipofectamine 3000 (Thermo Fisher Scientific, USA). Stable cell lines were selected for culture using 3 *μ*g/mL puromycin (Sigma, USA) for one week.

### 2.3. Quantitative Reverse Transcription Polymerase Chain Reaction (qRT-PCR)

Total RNA extraction was accomplished by TRIzol reagent (Invitrogen, USA), and NanoDrop 2000 system (Thermo Fisher Scientific, USA) was utilized for the detection of RNA concentration. cDNA transcription of miRNA and mRNA was done, miRNA with the miScript IIRT Kit (QIAGEN, Germany), and mRNA with the ipsogen RT Kit (QIAGEN, Germany) and PrimeScript RT Master Mix (TaKaRa, Japan). miRNA expression and mRNA expression were measured with the miScript SYBR Green PCR Kit (QIAGEN, Germany) and SYBR® Premix Ex Taq TM II (TaKaRa, Japan). Applied Biosystems®7500 Real-Time PCR Systems (Thermo Fisher Scientific, USA) was applied for qRT-PCR analysis. U6 spliceosomal small nuclear RNA (U6 snRNA) and *β*-actin were taken as internal controls.  Table 1 displayed the primer sequences. Differences in the relative level of miR-145-5p and HMGB3 mRNA were compared by 2^−ΔΔ*Ct*^.

### 2.4. Cell Counting Kit-8 (CCK-8) Assay

2 × 10^3^ cells/well were seeded into 96-well plates with 100 *μ*L DMEM containing 10 *μ*L FBS per well. The medium was changed with DMEM (100 *μ*L) plus CCK-8 (10 *μ*L, Beyotime, China) at a designated time point on indicated days, and cells were cultured for 2 h. Next, absorbance was read at 450 nm (optical density (OD)), and cell viability in each group was estimated using an average OD value.

### 2.5. Wound Healing Assay

Transfected BC cell line MDA-MB-231 and ZR-75-30 were plated into 6-well plates (1 × 10^6^ cells/well) with DMEM complete medium and 10% FBS. When reaching 80% of cell coverage, a 200 *μ*L sterile plastic tip was applied to scratch the surface of cells to create a line. Cell fractions were rinsed off with PBS. Cells were continuously cultured in medium without serum. At 0 h and 24 h, wounds were photographed by a phase-contrast microscope. Wound distance was measured to calculate the rate of wound closure at 24 h according to the formula hereinafter: wound healing rate = (the wound width of 0 h − the wound width of 24 h)/0 h wound width. This experiment was repeated independently 3 times.

### 2.6. Transwell Invasion Assay

Matrigel (356234, BD Company, USA) was dissolved at 4°C overnight, diluted with serum-free medium at 1 : 3, supplemented to the transwell chamber (8 *μ*m; Corning Inc., USA) with 50 *μ*L per well, and incubated for 30 min. The transfected cells (5 × 10^4^ cells/well) in FBS-free DMEM were plated in the upper chamber, and the lower chamber was added with DMEM to complete medium plus 10% FBS. Under standard culture conditions, cells were cultured for 24 h. Subsequently, a cotton swab was employed to remove cells on the membrane of the transwell chamber. Cells under the membrane were treated with 3 PBS washes, fixed with 4% paraformaldehyde solution for 30 min, and dyed with 0.1% crystal violet for 30 min. 5 fields were randomly chosen and the average number of invading cells in these fields were counted under a microscope.

### 2.7. Western Blot

RIPA buffer (Sigma, USA) plus phenylmethanesulfonylfluoride was applied to lyse cells and the BCA assay kit (Sigma, USA) to determine the concentration of total proteins. 10% SDS-PAGE was utilized for the separation of equivalent proteins (20 *μ*g) which were then transferred onto a PVDF membrane (Sigma, USA). 5% skim milk was utilized to seal the membrane for 1 h at room temperature. Next, the membrane was maintained with primary antibodies (rabbit anti-HMGB3 (ab72544, Abcam, UK), rabbit anti-E-cadherin (ab40772, Abcam, UK), rabbit anti-N-cadherin (ab76011, Abcam, UK), rabbit anti-vimentin (ab92547, Abcam, UK), and rabbit anti-*β*-actin (ab115777, Abcam, UK)) overnight at 4°C. Afterwards, the membrane was rinsed with PBST thrice each time for 10 min and was maintained with secondary goat anti-rabbit IgG H&L (ab205718, Abcam, UK) for 1 h under room temperature. The ECL kit (Solarbio, China) was applied for development. The ChemiDoc XRS Plus imaging analyzer (Bio-Rad, USA) was used for imaging. ImageJ software (NIH, USA) was utilized to analyze protein band gray values.

### 2.8. Dual-Luciferase Assay

miR-145-5p binding sites into the wild-type (WT)/mutant (MUT) 3′ untranslated region (3′UTR) of HMGB3 were synthesized and were then cloned into the pmirGLO vector (Generay, China) to obtain HMGB3-WT and HMGB3-MUT vectors, respectively. Cells were transfected with synthesized plasmids and miR-145-5p mimics/miR-145-5p inhibitor. Luciferase analysis was undertaken after 48 h transfection on the dual-luciferase reporter gene analysis system (Promega, USA) on the Fluoroskan Ascent Type 379 fluorescence plate reader (Thermo Fisher Scientific, USA). The standardized luciferase activity was reported as firefly luciferase intensity/Renilla luciferase intensity.

### 2.9. Flow Cytometry

1 × 10^6^ transfected cells were gathered for flow cytometry. After two washes with PBS, cells were collected, stained with the Annexin V-FITC/PI cell apoptosis detection kit (BD Biosciences, USA), detected by BD Accuri C6 Plus (BD Biosciences, USA), and analyzed by FlowJo software.

### 2.10. Analysis of Statistics

Data were processed using SPSS 22.0 and expressed as mean ± SD. Intragroup differences were analyzed by Student's *t*-test, while analysis of variance was applied for comparison among groups. The Kruskal Wallis test was utilized to analyze differences in HMGB3 expression in BC with different clinical features and subtypes. Kaplan-Meier was applied for survival analysis. Differences in the survival rate were tested via log-rank. *P* ≤ 0.05 was statistically significant. Samples in each group were plated in triplicate and each experiment was repeated 3 times.

## 3. Results

### 3.1. HMGB3 Expression Is Substantially High in BC Cells

Differential analysis was performed on mRNA expression data in TCGA. Then, we noted that the HMGB3 level was remarkably higher in BC tissues (Figure 1(a)). According to survival analysis, the HMGB3 high level was implicated in poor survival of BC patients (Figure 1(b)), especially Luminal A- (LumA-) type BC (Supplementary Figure (available here)). Besides, HMGB3 was significantly correlated with clinical features (T stage, N stage) of BC (Figure 1(c)). In addition, the HMGB3 level varied significantly in different subtypes of BC (LumA, LumB, HER2 enriched, basal like, and normal like) (Figure 1(d)). Next, the HMGB3 level in the human breast epithelial cell line and 4 BC cell lines was detected and it was displayed that HMGB3 mRNA and protein levels were markedly elevated in BC cells (Figures 1(e) and 1(f)). The above results indicated that in BC cells, HMGB3 expression remained at a notably high level. To dive deeper into the functional mechanism of HMGB3 in BC, MDA-MB-231and ZR-75-30 with the highest HMGB3 expression were utilized for the following experiments.

### 3.2. Altered HMGB3 Expression Affects BC Cell Proliferation, Invasion, Migration, Apoptosis, and EMT

To figure out the effect of HMGB3 in BC cells, HMGB3 was overexpressed in MDA-MB-231 cells and knocked down in ZR-75-30 cells and the corresponding control groups were constructed. qRT-PCR suggested that HMGB3 was substantially upregulated in the oe-HMGB3 group and downregulated in the si-HMGB3 group (Figure 2(a)). Additionally, overexpressing HMGB3 substantially promoted proliferative, invasive, and migratory properties of MDA-MB-231 cells. Knockdown of HMGB3 suppressed those properties of ZR-75-30 cells (Figures 2(b)–2(d)). Moreover, flow cytometry showed that overexpressing HMGB3 markedly downregulated the apoptotic level of MDA-MB-231 cells whereas silencing HMGB3 upregulated ZE-75-3P cell apoptosis (Figure 2(e)). The inverted microscope was utilized for observing the cell morphology of MDA-MB-231 cells. The elongated spindle mesenchymal cells increased after HMGB3 overexpression. The proportion of paving stone-like cells in ZR-75-30 cells increased after HMGB3 knockdown (Figure 2(f)). With the development of cancer, the elevated expression of mesenchymal cell markers like vimentin and N-cadherin indicates that cancer cells are undergoing epithelial-mesenchymal transition (EMT). The Western blot result displayed that protein expression of E-cadherin (epithelial marker) could be downregulated but protein expression of N-cadherin and vimentin could be upregulated by overexpressed HMGB3. HMGB3 overexpression significantly promoted the EMT process of MDA-MB-231 cells (Figure 2(g)). In conclusion, overexpressed HMGB3 facilitated malignant phenotype progression of BC cells but the knockdown of HMGB3 had an opposite effect.

### 3.3. MiR-145-5p Is Predicted as an Upstream Regulatory miRNA of HMGB3 in BC Cells

To study upstream functional mechanism of HMGB3 in BC cells, EdgeR was applied for differential analysis and 74 differential miRNAs were acquired (55 upregulated miRNAs and 19 downregulated miRNAs) (Figure 3(a)). Next, differentially downregulated miRNAs were overlapped with target miRNAs predicted by databases to obtain miR-145-5p (Figure 3(b)). Notable negative correlation was represented between HMGB3 and miR-145-5p as well (Figure 3(c)). In comparison to normal breast tissue, BC tissue had a remarkably lower miR-145-5p level (Figure 3(d)). Then, miR-145-5p in 4 BC cell lines was also shown to have a significant downregulation by qRT-PCR (Figure 3(e)). In summary, miR-145-5p showed a low-level expression in BC cells, which may restrain BC cell progression.

### 3.4. miR-145-5p Targets HMGB3 in BC

By using bioinformatics, it was discovered that miR-145-5p and HMGB3 had a binding relationship (Figure 4(a)). Thereafter, their binding was proved via dual-luciferase analysis and it was elucidated that overexpressing miR-145-5p or inhibiting miR-145-5p restrained or stimulated luciferase activity of cells with WT HMGB3 3′UTR, respectively, but for MUT HMGB3 3′UTR, there was no effect on it (Figure 4(b)). Next, the HMGB3 mRNA level in MDA-MB-231 and ZR-75-30 cell lines in the transfection groups was measured by qRT-PCR. The result demonstrated that HMGB3 mRNA level was notably decreased in miR-145-5p overexpressed cell lines, but it showed a marked increase in miR-145-5p inhibitor cells (Figure 4(c)). As revealed via Western blot, upregulating miR-145-5p remarkably reduced HMGB3 protein expression whereas inhibiting miR-145-5p noticeably increased the HMGB3 protein level (Figure 4(d)). All the above results presented that miR-145-5p targeted HMGB3 and suppressed its level in BC cells.

### 3.5. miR-145-5p Inhibits BC Cell Proliferation, Migration, Invasion, and EMT and Promotes Apoptosis via Negatively Regulating HMGB3

The MDA-MB-231 cell line with overexpressed HMGB3 or miR-145-5p alone and simultaneously overexpressed HMGB3 and miR-145-5p were established. The miR-145-5p inhibitor and si-HMGB3 were transfected to ZR-75-30 cells. qRT-PCR analysis demonstrated that HMGB3 expression was substantially lower in the miR-mimic + oe-NC group when with a contrast to that in the NC group. Compared with those of miR-145-5p mimic + oe-HMGB3 and miR-mimic + oe-NC cells, the HMGB3 mRNA level was elevated. But it was hindered in the miR-145-5p mimic + oe-HMGB3 group compared with that in the miR-NC + oe-HMGB3 group. Likewise, simultaneously inhibiting miR-145-5p and HMGB3 recovered the promoting effect of the miR-145-5p inhibitor on HMGB3 expression (Figure 5(a)). By observing cell morphology, overexpressed miR-145-5p elevated the proportion of paving stone-like cells (Figure 5(b)). As suggested by Western blot, overexpressing miR-145-5p alone substantially suppressed HMGB3, N-cadherin, and vimentin protein levels, while elevating E-cadherin protein expression, while overexpressing HMGB3 as well could recover these effects. Inhibition of miR-145-5p and HMGB3 simultaneously restored the promoting effect of the miR-145-5p inhibitor on EMT of BC cells (Figure 5(c)), which further denoted that overexpressing miR-145-5p counteracted the facilitating impact of HMGB3 on protein expression and the EMT process of cancer cells. Additionally, overexpressing miR-145-5p remarkably restrained the proliferative, invasive, and migratory properties of BC cells, while overexpressing HMGB3 simultaneously could offset such effect. Simultaneous inhibition of miR-145-5p and HMGB3 expression reversed the promoting effect of knockdown of miR-145-5p on malignant progression of BC cells (Figures 5(d)–5(f)). Additionally, it was also identified by flow cytometry that transfecting miR-145-5p could noticeably stimulate BC cell apoptosis while simultaneously overexpressing miR-145-5p, and HMGB3 recovered such effect. Simultaneously inhibiting miR-145-5p and HMGB3 rescued the repressive effects of the miR-145-5p inhibitor on BC cell apoptosis (Figure 5(g)). These results concluded that miR-145-5p downregulated HMGB3 expression to suppress malignant progression of BC cells.

## 4. Discussion

In recent years, major progress had been made in researching BC in biology with the improved diagnostic technology and newly developed targets. This study was also made in researching BC and manifested that miR-145-5p downregulated HMGB3 expression to suppress malignant progression of BC cells.

Currently, HMGB3 protein has shown substantial effect on the development of BC [13, 14]. High-level HMGB3 is usually discovered in BC and it exerts a cancer-promotive role in cancer [22, 23]. Much literature so far verifies that HMGB3 may be a biomarker of several cancers. It has already been shown that HMGB3 had a targeting relationship with miR-145 in non-small cell lung cancer [24]. In BC cells, HMGB3 is upregulated and its silencing impairs cell proliferation *in vitro* and *in vivo* [15]. It is worth noting that the study of Li et al. [25] manifested that enforced HMGB3 expression accelerates bladder cancer cell proliferation and pertains to poor survival outcomes, which is consistent with our study results. This study demonstrated the highly expressed HMGB3 in BC cells, and it could enhance proliferation, migration, invasion, and the EMT process of tumor cells, while inhibiting cell apoptosis.

This study predicted by bioinformatics analysis showed that miR-145-5p had a targeting relationship with HMGB3. Several studies have discovered that various cancers have remarkably low-level miR-145-5p expression which can inhibit the advancement of bladder cancer [26], non-small cell lung cancer [27], and gastric cancer cells [28]. Similarly, we found the significantly low-level miR-145-5p expression in BC cells and the dual-luciferase assay demonstrated that there was indeed a targeting relationship between HMGB3 and miR-145-5p. We also discovered that miR-145-5p was capable of negatively regulating the expression of HMGB3. Cell function experiments showed that overexpressed miR-145-5p could reverse the promoting effect of overexpression of HMGB3 on proliferation, invasion, and migration of tumor cells.

In summary, these findings demonstrated the high HMGB3 in BC, which was closely bound up to the poor prognoses of BC patients. miR-145-5p, by targeting HMGB3, could inhibit the proliferative, invasive, and migratory abilities and facilitated apoptosis of BC cells. This study reveals that the miR-145-5p/HMGB3 signaling axis is a new network that regulates the advancement of BC cells, which provides a prospective strategy for the diagnosis and treatment of BC.

## Figures and Tables

**Figure 1:** HMGB3 expression is substantially high in BC cells. (a) Boxplot of HMGB3 expression in healthy breast tissues and BC tissues (comparison between two groups: *P* < 2*e* − 16). (b) Survival analysis of HMGB3 expression on BC patient's prognosis (comparison between two groups: *P* = 1.042*e* − 02). (c) Correlation between HMGB3 and BC clinical features (T stage, N stage, asterisk indicates statistically significant differences, and *P* < 0.05). (d) Relationship between HMGB3 expression and BC subtypes (asterisk indicates statistically significant differences and *P* < 0.05). (e, f) HMGB3 mRNA and protein levels in human breast epithelial cell line MCF-10A and BC cell lines MDA-MB-468, MDA-MB-231, T47D, and ZR-75-30. Results were presented as mean ± SD. Log-rank test was utilized for survival analysis. Correlation between HMGB3 and clinical features with different subtypes of BC was analyzed by the Kruskal-Wallis test. The others were statistically analyzed by Student's *t*-test. Samples in each group were plated in triplicate. ^∗^*P* < 0.05.

**Figure 2:** Altered HMGB3 expression affects BC cell proliferation, invasion, migration, apoptosis, and EMT. (a) Transfection efficiency of cells in each group. (b) BC cell proliferation. (c) BC cell invasion (magnification: 100x; migrating cell numbers were the average value of 5 random fields). (d) Migratory ability of BC cells (magnification: 40x; wound healing rate = (0 h wound width − 24 h wound width)/0 h wound width). (e) Apoptotic rate of BC cells. (f) Morphology changes of cells were detected by an inverted microscope. (g) Protein expression of E-cadherin, vimentin, and N-cadherin in BC cells. Student's *t*-test was employed for statistics. Samples in each group were plated in triplicate. The experiments were repeated thrice. ^∗^*P* < 0.05.

**Figure 3:** Low level of miR-145-5p in BC cells. (a) Volcano plot of differential miRNAs in the TCGA-BRCA dataset (red: 55 upregulated miRNAs; green: 19 downregulated miRNAs). (b) Intersection between predicted upstream regulatory genes of HMGB3 and differentially downregulated miRNAs. (c) Correlation between HMGB3 and miR-145-5p (comparison between two groups: *P* = 1.736*e* − 54). (d) Boxplot of miR-145-5p expression in normal and tumor groups (comparison between two groups: *p* < 2*e* − 16). (e) miR-145-5p level in normal and BC cell lines. Results were shown as mean ± SD. Data analysis was completed by Student's *t*-test. Samples in each group were plated in triplicate. ^∗^*P* < 0.05, compared with the corresponding NC group.

**Figure 4:** miR-145-5p targets HMGB3 in BC cells. (a) Predicted binding sites between miR-145-5p and HMGB3. (b) Luciferase activity of cells in the transfection groups. (c) Level of HMGB3 mRNA of cells in treatment groups. (d) Level of HMGB3 protein of cells in treatment groups. Results were shown as mean ± SD. Data were analyzed via Student's *t*-test. Samples in each group were plated in triplicate. 3 repetitions were carried out for each experiment. ^∗^*P* < 0.05, compared with the corresponding NC group.

**Figure 5:** miR-145-5p suppresses BC cell phenotype progression through targeting HMGB3. (a) Level of HMGB3 mRNA of cells in the groups. (b) Changes of cell morphology as detected by an inverted microscope. (c) Protein levels of E-cadherin, vimentin, N-cadherin, and HMGB3 cells in treatment groups. (d) Cell proliferation in treatment groups. (e) Cell invasion in treatment groups (magnification: 100x; migrating cell numbers are the average value of 5 random fields). (f) Cell migration in transfection groups (magnification: 40x; wound healing rate = (0 h wound width − 24 h wound width)/0 h wound width). (g) Apoptotic level of cells in transfection groups. Data were analyzed via Student's *t*-test. Samples in each group were plated in triplicate. Each assay was performed 3 times. ^∗^*P* < 0.05.

**Table 1:** Primer sequences used in the assay.

Gene	Primer sequences (5′→3′)
miR-145-5p	F: GCCGAGGTCCAGTTTCCCA
	R: CTCAACTGGTGTCGTGGA

U6 snRNA	F: CTCGCTTCGGCAGCACA
	R: AACGCTTCACGAATTTGCGT

HMGB3	F: GACCAGCTAAGGGAGGCAA
	R: ACAGGAAGAATCCAGACGGT

*β*-Actin	F: CACCATTGCAATGAGCGGTTC
	R: AGGTCTTTGCGGATGTCCACGT

## Data Availability

The data used to support the findings of this study are included within the article.

## Supplementary Materials

Supplementary Materials Supplementary Figure: the relationship between HMGB3 expression and the prognosis of different subtypes of BC. A–E Analysis of HMGB3 expression and the survival of basal-like-type, Her2E-type, LumA-type, LumB-type, and normal-like-type BC patients, respectively. Survival analysis was performed using the log-rank test.
